The article "Construction of a Prediction Model for Distance Education Quality Assessment Based on Convolutional Neural Network" was published in 2022. Journal: Comput Intell Neurosci.

# Construction of a Prediction Model for Distance Education Quality Assessment Based on Convolutional Neural Network

**DOI:** 10.1155/2022/8937314

**Published:** 2022-09-05

**Authors:** Peizhang Wang

**Affiliations:** School of Management, Anhui Science and Technology University, Chuzhou, Anhui 233100, China

## Abstract

This paper introduces the principles and operation steps of convolution and pooling of convolutional neural networks in detail. In view of the shortcomings of fixed sampling points and single receptive field in traditional convolution and pooling forms, deformable convolution and deformable pooling are introduced to enhance the network's ability to adapt to image details and large displacement problems. The concepts of warp, loop optimization, and network stack are introduced. In order to improve the optimization performance of the algorithm, three subnetwork structures and stack models are designed, and various methods are used to improve the prediction accuracy of distance education quality assessment. In order to improve the accuracy and timeliness of education quality assessment, this paper proposes a distance education quality assessment model based on mining algorithms. The prediction index is selected by the improved BP neural network. It is required to establish the input layer node as the input vector based on the number of data sources since the input layer is used for data input. The neural network is trained with a quarter of the mining data, and the mining algorithm is further trained with network error trials. A fuzzy relationship matrix is created based on the assessment of teaching quality's hierarchical structure. This leads to the conclusion of the fuzzy thorough evaluation of the effectiveness of distant learning. Experiments show that the proposed model has an average accuracy of 96%, the average teaching quality modeling time is 25.44 ms, and the evaluation speed is fast.

## 1. Introduction

Distance education is a type of education that transmits courses to one or more students away from the campus using a variety of media for systematic teaching and communication. Nowadays, remote learning refers to learning that is done by computer technology, both real-time and nonreal-time, audio, and video (live or video). Modern distant learning is a brand-new educational format modified for use with contemporary information technology [1]. In May 2020, the Ministry of Education revealed at a press conference that online teaching will become the new normal after resumption of school in colleges and universities. Our country's higher education enterprise has obtained the rapid development, accepted the higher education, and the object to have the significant increase. The number of university teachers has also increased significantly, and the effects of higher education have had a significant impact on the country's economic development [2, 3]. College teachers are both educators and researchers, and the requirements for teachers have reached a new height [4–6].

The article "Construction of a Prediction Model for Distance Education Quality Assessment Based on Convolutional Neural Network" was published in 2022. Journal: Comput Intell Neurosci.

For neural networks, people often hope that the established network model can focus on the most representative feature information in a certain field, so as to avoid the problem of overfitting and improve the performance of the network model. The scale is getting bigger and bigger, and there are more and more internal parameters, and the problem of information overload caused by it also needs to be solved urgently. By introducing the attention mechanism, the above two types of problems can be solved, focusing on the most useful information for the task among the many information, while reducing the attention to the secondary information and eliminating irrelevant information, which can improve the accuracy of the model and avoid information overload question.

The commonly used attention models include temporal attention and spatial attention, and the specific function of attention can be divided into hard attention mechanism and soft attention mechanism. The hard attention mechanism means that in front of multiple objects or features, only a weight value of 1 is taken, while the others are 0, that is, only one point is concerned; while the soft attention mechanism is to take the weight of multiple objects or features. The value setting range, such as [0, 1], is only divided into primary and secondary instead of partial generalization, so the soft attention mechanism is the most commonly used attention mechanism. Since the advantages of the attention mechanism are applicable to regular data, it is most widely used in the research of image processing and computer vision.

In order to systematize the management, office automation and informationization of teacher evaluation in colleges and universities, it is necessary to conduct research and discussion in all aspects. The content and system of teacher assessment, as well as data processing and analysis of assessment results, need further study. How to make comprehensive use of pedagogy, statistics, information network technology, and computer technology to design a high-efficiency and high-quality system is an important content of teacher management and evaluation. This research suggests a mining algorithm-based methodology for evaluating the quality of distant education in order to increase its accuracy and efficacy.

## 2. Method

### 2.1. Data Mining Algorithms

It has the advantage of allowing mining computations to be performed using data stored in the current information system, and to encapsulate complex statistical techniques and mining algorithms through computer application programs. Even without mastering these techniques, the same function can be accomplished, thereby focusing more on the problem to be solved [7, 8]. In light of the aforementioned factors, this work intends to incorporate data mining technology into the field of teaching assessment and investigate a model for evaluating the quality of distant education.

The article "Construction of a Prediction Model for Distance Education Quality Assessment Based on Convolutional Neural Network" was published in 2022. Journal: Comput Intell Neurosci.

At present, artificial neural networks are a fast growing area of frontier research that have profound effects on cognitive science, information technology, and artificial intelligence in computer science. Additionally, it is crucial for data mining [9, 10]. For a very long time, BP neural networks have been applied in data mining. However, the modified approach has to be improved because it has a problem with local minimization.

The selection of the predictive indicator, which is based on the performance of the students in distance education, is the first stage in building the improved BP neural network model. Next, the vectors for the output and input are created [11, 12]. Input layer nodes must be set as input vectors in accordance with the amount of data sources since enter layer is used to input data.  Table 1 outlines the procedures for calculating the number of data sources.

The excitation function of the input layer node is as follows:

(1) $$\begin{array}{c} k\left(v\right)=\frac{1}{\exp\left(-\beta \right)v^{4}}. \end{array}$$

Among them, *k*(*v*) represents the activation function of the input layer node. *v* represents the function argument. *β* represents the slope control parameter.

The neuron corresponding to the input layer is the input vector. The following formula can be used to determine the output vector:

(2) $$\begin{array}{c} O_{i}=k\left(v\right)\cdot f{\left(\sum_{i=1}^{n}W_{i}\theta_{i}\right)}^{2}, \end{array}$$

where *O*_*i*_ represents the output of the output vector. *W*_*i*_ represents the weight of the output node. *θ*_*i*_ represents the threshold of the output layer.

Then, for the improved BP neural network, choose the number of layers or adjust the number of neurons in the hidden layer. Then, choose the corresponding hidden layer nodes, that is, begin to invest in a few hidden layer nodes [13, 14]. Then gradually increase the number of invested nodes until the number of nodes is more manageable. This procedure must be tested. The hidden layer node's corresponding output formula is as follows:

(3) $$\begin{array}{c} y_{i}=O_{i}f\left(\sum_{j=1}^{n}w_{i}{\;}_{j}x_{j}-\theta_{i}\right), \end{array}$$

where *y*_*i*_ represents the corresponding output of the hidden layer node. *w*_*i*_*j*__ represents the corresponding network weight of the hidden layer. *x*_*j*_ stands for input node.

The article "Construction of a Prediction Model for Distance Education Quality Assessment Based on Convolutional Neural Network" was published in 2022. Journal: Comput Intell Neurosci.

Using a quarter of the mining data, that is, training samples, to test and improve the BP neural network, first put eight neurons, and then increase to fifteen, and conduct tests, respectively [15].  Figure 1 displays the specific training results. Choose the number of neurons that corresponds to the best combination of training time and training error.

According to the above table, when the number of neurons is 15, the error can be kept to a minimum.

On this basis, different training functions are used to detect network errors, and a new BP neural network model is presented. A correction algorithm is used to optimize the design of the BP neural network based on the experimental data [16, 17]. Tests for network failures are shown in Table 2.

Choose lm to improve the BP neural network based on the results in the preceding table. And, based on the results in Tables 2 and 3, a three-layer improved BP neural network model is built. The model's network structure is 4, 15, and 1, with a total of four input nodes [18–20]. There is one output node and fifteen hidden nodes.

(4) $$\begin{array}{c} \left\{\begin{array}{c} f\left(L^{\left(k+1\right)}\right)=\text{min}f{\left(X^{\left(k\right)}+S\left(L^{\left(k\right)}\right)\right)}^{2}\eta^{\left(k\right)},\\ L^{\left(k+1\right)}=L^{\left(k\right)}+\eta^{\left(k\right)}S\left(L^{\left(k\right)}\right). \end{array}\right) \end{array}$$

Among them, *L*^(*k*)^ represents the threshold of the network and the vector of all values. *S*(*L*^(*k*)^) represents the search direction of the space vector formed by each function component in *X*. *η*^(*k*)^ stands for the minimum step size.

### 2.2. A Model for Evaluating the Quality of Distance Learning

A system of excellent teaching quality evaluation indexes must have the qualities of authenticity, specificity, and convenience.  Table 3 summarizes and categorizes the elements of all teaching quality evaluation systems, displaying a set of comprehensive, multifaceted, and multilevel three-dimensional evaluation index systems.

*r*_*ij*_(*i*=1,2, ⋯, *m*; *j*=1,2, ⋯, *n*) describes the result of the *i*th factor of the teacher being evaluated since the first factor and establishes the following fuzzy evaluation matrix:

(5) $$\begin{array}{c} R=\left[\begin{array}{cccc} r_{11} & r_{12} & \cdots & r_{1n}\\ r_{21} & r_{22} & \cdots & r_{2n}\\ \vdots & \vdots & \vdots & \vdots \\ r_{m1} & r_{mw} & \cdots & r_{mn} \end{array}\right], \end{array}$$

*S*=(*s*_1_, *s*_2_, ⋯, *s*_*m*_) is a very important set of B. When both *R* and S are known, both can be blurredly transformed to obtain model *W*=(*R* × *S*)=(*d*_1_, *d*_2_, ⋯, *d*_*n*_)[18, 21, 22].

The article "Construction of a Prediction Model for Distance Education Quality Assessment Based on Convolutional Neural Network" was published in 2022. Journal: Comput Intell Neurosci.

Construct a comprehensive evaluation factor set *Z*.

Many different elements are frequently included in an excellent teaching quality rating method. It will be challenging to analyze, nevertheless, if the criteria to be taken into account are overly extensive. There is established a set of evaluation criteria for thorough consideration: *X* = “The lesson preparation is thorough, and the teaching style is appropriate.” The emphasis in the classroom is on helping students understand; engaging in classroom discussion; and energizing the learning environment. Be tough with yourself and set an example for kids. Teach students according to their aptitude. Focus on ability training. Care for students and be genuinely appreciated by them”.

Build an evaluation set Y.

The evaluation set can serve as a reflection of a teacher's instructional ability. The evaluation set commonly divides teachers' teaching levels into three categories: “outstanding,” “good,” “average,” and “bad.” As a result, each level contained in Y can only have values inside a specific range during the actual evaluation. The text range can be set as [50, 100] and divided into four decreasing intervals based on the analysis mentioned above. If the obtained score falls within [80, 100], it can be set at 90, designating the teacher as having “outstanding” teaching status. If the obtained score falls within [70, 90], it can be set to 80, indicating that the teacher's performance as a teacher is “good.” The teacher's teaching status may only be described as “average” if the obtained score is placed in the range [60, 80], since that score's median value is 70. If the obtained score falls between [50 to 70], the score might be set to 60, indicating that the teacher's teaching condition is “poor,” or not good. In reality, though, fractional division is based on the middle value of each fractional interval, and the parameter column vector can be adjusted to *Y* = [90, 80, 70, 60].

Establishing the evaluation factor set's weight set is crucial since each factor holds a unique key location inside the evaluation factor set, meaning that each factor's weight is different. How to assess the accuracy of evaluation results by judiciously allocating the weight of each component. The Delphi technique is a reliable system for determining weight. The main principle of the Delphi method is to collect anonymous expert opinions, analyze them, and then transmit them to other experts in a similar manner.

The article "Construction of a Prediction Model for Distance Education Quality Assessment Based on Convolutional Neural Network" was published in 2022. Journal: Comput Intell Neurosci.

Build a fuzzy relationship matrix.

Based on teachers' daily behavior in a variety of criteria, all assessors provide objective evaluations. By using induction and sorting, a fuzzy relationship matrix *R* is created, and the possibility measure is then derived. If there are 200 people participating in the evaluation of a certain aspect of teacher evaluation, of which 140 were rated as “excellent”, 40 were rated as “good”, 20 were rated as “general”, the probability of the result being “excellent” is 140/200 = 0.7. The probability of good is 40/200 = 0.2. The probability of “general” is 20/200 = 0.1. The probability of “poor” is 0/200 = 0. Obtain the results of the fuzzy through evaluation.

(6) $$\begin{array}{c} W=\left(R\times S\right)=\left(d_{1},d_{2},d_{3},d_{4}\right). \end{array}$$

The value obtained by using *S*=(*W* × *V*)=90*∗d*_1_+80*∗d*_2_+70*∗d*_3_+60*d*_4_ can serve as the teacher being evaluated's final assessment score. The range in the assessment set Y allows one to determine the teacher's teaching quality rating.

### 2.3. Overall Architecture of Convolutional Neural Network

The network model in this paper is optimized and improved based on the basic model of the convolutional neural network, including the feature extraction part, the feature fusion part, and the final optical flow output part. The process is shown in Figure 2.

The function of the feature extraction module is to extract the spatial information features of two adjacent frames in a continuous image sequence. It is mainly composed of a deformable convolutional layer and a traditional square convolutional layer. Its input is the adjacent two frames of RGB images I1 and I2. Two branches with the same structure and independent parameter weights extract the spatial features of the two frames to ensure that the feature dimensions of the output are consistent; the improvement of this part lies in the introduction of a deformable convolution layer, compared with the existing traditional square convolution layer. The composed convolutional neural network feature extraction module can better extract the image detail features of adjacent frames and improve the ability to capture large displacements, so as to solve the problems of large displacements and image detail rendering in optical flow prediction.

The feature fusion part can fuse the spatial features of two deep adjacent frames extracted from continuous image sequences into one feature, and calculate the correlation between the two frame features at the same time, which is mainly composed of a convolution layer based on the channel attention mechanism. The importance of each channel is calculated, and additional weights are added to each channel to reconstruct the features; the improvement of this part is reflected in the feature fusion method using the attention mechanism. Compared with the existing matching-based fusion method, the correlation between two frames can be better calculated. The key to optimizing the occlusion problem lies in the calculation of deep feature correlation. Therefore, the improvement of this part can, in principle, enhance the network in a targeted manner.

The article "Construction of a Prediction Model for Distance Education Quality Assessment Based on Convolutional Neural Network" was published in 2022. Journal: Comput Intell Neurosci.

In order to improve the prediction effect of the model for the problems of occlusion, large displacement, and image detail rendering between consecutive frame images, and at the same time to ensure its universality, it has excellent accuracy for various images and motion forms. Using the strategy of cyclic optimization, through the improvement of the DANet-S network structure, a total of three subnetworks with different characteristics are designed, and then multiple subnetworks are connected, and the output optical flow of each layer of network and the actual optical flow are calculated through Warp. The loss of the flow enables the lower network to focus on learning this part of the loss, thereby improving the prediction accuracy of the method in this paper.

### 2.4. Interframe Feature Association Layer Based on Attention Mechanism

The optimization of the feature fusion part of the convolutional neural network for optical flow prediction is the key to solving the occlusion problem. Shallow-level spatial feature extraction cannot accurately characterize the occluded part of the image. It is necessary to calculate the correlation between two adjacent frames in the deep-level feature, so as to find the motion and correspondence of the occluded part in the two images.

The matching mechanism employed by the model is difficult to capture the complex motion between adjacent frames. The attention mechanism is suitable for the convolutional neural network to solve targeted and focused image problems. Therefore, in order to better calculate the correlation between the spatial features of two adjacent frames, we improve the network model's ability to deal with the problem of image object occlusion. In this paper, a feature correlation layer based on the channel attention mechanism is designed. Through this module, the correlation of the features of two adjacent frames is calculated, and the fusion reconstruction is performed to enhance the network's processing ability to the occlusion problem.

The attention mechanism is like when the human eye or a camera observes or shoots an object, its focus must be focused on the object of interest, while ignoring other objects or backgrounds. It is blurred, and for an intelligent human brain, it will even directly filter out irrelevant information such as the background, so as to eliminate interference; similarly, when the target object changes, its attention will also shift and focus on another target. This means that the spatial distribution of attention or attention points is different, and the importance of each object or background is proportional to the distribution of attention; in terms of time, it is impossible for every sentence of a piece of news to have the same amount of attention. Equally important, some segments are the key information of the reported event, while some segments are modifiers that are not related to the event. The distribution of these segments in time is different, which also leads to the listener's attention on the time series.

The article "Construction of a Prediction Model for Distance Education Quality Assessment Based on Convolutional Neural Network" was published in 2022. Journal: Comput Intell Neurosci.

When processing text, the input sentence is composed of multiple words, and the words have different grammatical status and different importance in understanding the meaning of the sentence. The Decoder framework treats these words equally, extracts semantic information in the same way for each word, then converts it into the output word, and then combines it into a complete sentence. When dealing with image data or image features, this framework also treats each region of the image or feature spatial distribution as “the same”, and the next step is processed with the same weight for information in different spatial or channel positions.

Education quality evaluation is based on certain educational quality standards and goals, and relies on scientific educational evaluation methods and methods to make value judgments on the development status and influence of the evaluation object. Evaluation can provide reliable information for human development and education decision-making and assist education decision-makers in choosing the best strategies. The distance education quality assessment mode based on convolutional neural network is shown in Figure 3.

## 3. Experiment and Analysis

The purpose of this experiment is to explore the application effect of data mining methods in the evaluation of college education quality. This paper selects three types of distance online teaching platforms with prominent styles for testing: the first type of distance online teaching platform is characterized by high quality and relatively rich course content, and the instructors are experienced teachers. For example, NetEase Open Course, MOOC., which we call the content class. The second category is characterized by strong interactivity and timely feedback, usually live teaching, such as QQ groups and Tencent conferences. This article calls it the interactive category. The third type of platform is compatible with both and meets a certain degree of interactivity. It can record live courses and has playback functions, such as Tencent Classroom and DingTalk Live. This article calls them compatible classes.

The article "Construction of a Prediction Model for Distance Education Quality Assessment Based on Convolutional Neural Network" was published in 2022. Journal: Comput Intell Neurosci.

The users of the online teaching platform are relatively fixed. This paper randomly selects 100 teachers and students for evaluation by visiting 10 colleges and universities in a province and sending emails to users of the online teaching platform. 220 evaluation samples were scored by 100 users, and the specific distribution of their identity, gender, education level, and subject area is shown in Table 4. It can be seen from the distribution that the survey sample is representative to a certain extent and can better evaluate the use of the online teaching platform.

This paper uses the methods of Reference [5] and Reference [6] as the control group to verify the three methods to evaluate the quality of distance teaching of teachers in the 10 universities mentioned above.

### 3.1. The Accuracy of Distance Teaching Quality Assessment

The accuracy of distance teaching quality assessment of each university is counted, and the results are shown in Figure 4.

We analyze the results of the accuracy rate of teaching quality evaluation in Figure 1:

1. The teaching quality evaluation mistake is the biggest, and the approach in Reference [5] has an average evaluation accuracy of 85%. This is due to the fact that its parameters are chosen at random, making it impossible to develop an evaluation model that captures the intricate and ever-changing aspects of teaching quality. As a result, teaching quality assessment results in many overfitting points and has the worst teaching quality assessment effect.
2. The average accuracy of the distance teaching quality assessment method in Reference [6] is 90%, and the teaching quality assessment error is smaller than the standard BP neural network. This is because the support vector machine is introduced, and a better teaching quality evaluation model than the standard BP neural network is established, which can effectively describe the complex and changing characteristics of teaching quality. Due to the existence of some underfitting points in teaching quality evaluation, the evaluation effect needs to be further improved.
3. The two competing approaches of distant mathematics teaching quality evaluation accuracy are far from the average teaching quality evaluation accuracy of 96 percent used in this paper. This is because the model in this paper introduces the BP neural network to select the predictor, and uses a quarter of the mining data to train the neural network, and further trains the mining algorithm through the network error test. Therefore, an evaluation model that can adjust the complex characteristics of optimal educational change in an overly precise manner is developed. The model effectively improves the evaluation effect of distance teaching quality.

The article "Construction of a Prediction Model for Distance Education Quality Assessment Based on Convolutional Neural Network" was published in 2022. Journal: Comput Intell Neurosci.

### 3.2. Efficiency of Distance Teaching Quality Assessment

In practice, with the continuous increase of data, the evaluation of teaching quality in colleges and universities has also received increasing attention. In order to analyze the validity of university education quality evaluation, the modeling time of university teaching quality under different modes was calculated. The results are shown in Figure 5.

It can be considered from Figure 2 that the suggest time of the approach in Reference [5] is 62 ms, and the suggest time of the educating high-quality modeling in Reference [6] is 39.27 ms. The average teaching quality modeling time of this method is 25.31 ms. The comparison results show that the approach described in this paper's teaching quality modeling time is significantly reduced, and the effectiveness of teaching quality evaluation in remote institutions is enhanced.

### 3.3. Prediction Results and Analysis of Distance Education Quality Assessment

The model in this paper is mainly built on the public server of the research group. The processor of the deep learning server uses Intel Core I7-5960X (main frequency: 3.0 GHZ), the model of the graphics accelerator is NVIDIA GeForce GTX1080Ti, and the operating system is Linux (Ubuntu version is 18.04), the Cuda version is 9.0, the program is built and trained under the Pytorch 0.4.1 framework, and the main programming languages used are python and linux scripting languages.

The network is trained and adjusted in the form of supervised learning, and the average end-point error of the predicted optical flow and the real optical flow is used as the loss function of the network backpropagation, that is, the comparison between the ground truth from the dataset and the image after the predicted optical flow interpolation. The data set and strategy used for training will greatly affect the network performance.

The prediction robustness and *F*1 value of the distance education quality assessment of the three algorithms are shown in Figures 6 and 7, respectively.

### 3.4. General Analysis of Distance Teaching Quality Assessment

Ten courses from a university were chosen as the test items, and their distance teaching quality assessment accuracy and modeling time were tallied in order to investigate the generality of the data mining algorithm's distance teaching quality assessment model.  Table 5 presents the outcomes.

The article "Construction of a Prediction Model for Distance Education Quality Assessment Based on Convolutional Neural Network" was published in 2022. Journal: Comput Intell Neurosci.

As shown in Table 5, the model in this research not only produces highly accurate findings for the quality evaluation of distance teaching, but also that the evaluation speed is rather quick. The approach can be used to evaluate the effectiveness of teaching in colleges and universities in a way that is practical and applicable.

## 4. Discussion

In this paper, deformed convolution, pooling, and channel attention mechanisms are introduced into the convolutional neural network model. In principle, the feasibility of deformed convolution and pooling to solve complex motion problems is analyzed, and a feature extraction part based on deformed convolution is established. Furthermore, the superiority of the attention mechanism in the field of optical flow prediction is clarified, which realizes the feature association layer based on the channel attention mechanism.

The initial parameters of the network model in this paper are uniformly set through the same initialization method. The network level and cascade method are all based on experience and experiments, and lack theoretical support. This is also the current deep learning in the network structure. A series of related theories should be established to solve common problems in parameter optimization, and there should be corresponding standards for solving problems of different scales and types.

The deformable convolution and channel attention mechanisms used in the model in this paper have targeted optimization for issues such as occlusion, large displacement, and image detail presentation in the field of optical flow prediction, but other related issues are not covered. For the prediction of single-frame image optical flow, multitarget motion and weak texture, no effective solutions have been proposed. These issues should also be the focus of future research.

Because the convolutional neural network has a certain randomness in the training convergence process, especially when the data set is not sufficient, it is easy to lead to local convergence, and the global optimal solution cannot be obtained, which leads to poor stability of network training. The proposed optical flow prediction network model introducing deformable convolution and channel attention mechanism also suffers from similar problems. Therefore, it is necessary to conduct more in-depth research and exploration on the training and convergence methods of the network, and improve the stability and accuracy of network training from the aspects of network structure, propagation mode, basic composition, and optimization training strategy. This has important practical significance for the research and application of optical flow prediction algorithms, and has more practical significance for the development of neural networks, deep learning and artificial intelligence, and is the next development direction of these fields.

The article "Construction of a Prediction Model for Distance Education Quality Assessment Based on Convolutional Neural Network" was published in 2022. Journal: Comput Intell Neurosci.

Teachers' teaching and research work is the guarantee of school education quality. In the research work, teachers evaluate the teachers who have listened to the class, point out their shortcomings, and praise their strengths. The teachers who evaluate the class not only reflect on their own shortcomings in the process of pointing out the teachers who are listening to the class but also can improve their own teaching. Teachers express their opinions in teaching and research activities, and different teachers have different understanding levels of the same content. An exchange between different teaching methods, discussing different courses using different teaching methods can improve teachers' teaching ability, thereby improving their teaching ability.

## 5. Conclusion

The basic concepts and principles of the attention mechanism are introduced, the structural flow of the Encoder-Decoder framework is analyzed in detail, and the application form of the attention mechanism in the convolutional neural network is expounded. This paper proposes a feature correlation layer based on the channel attention mechanism, which improves the network adjustment and adaptation ability and correlation calculation ability without increasing too much computational cost. The cause of teaching reform in colleges and universities must be advanced day by day due to the ongoing advancement of the times. How to raise teaching standards is the most crucial challenge in the reforming process. We can only introduce exceptional potential to society by reforming colleges and institutions. In order to develop a mathematical model for assessing the effectiveness of distant education, this research makes use of data mining technology. After the number of samples is determined, the BP neural network based on 1/4 mining is used for training, and the network error experiment is carried out. On this basis, the quality of distance education is evaluated by fuzzy correlation matrix. According to experimental data, the model's average assessment accuracy is 96 percent, the average teaching quality modeling time is 25.44 milliseconds, and the evaluation speed is higher. The model developed in this research has certain advantages over the other models in terms of evaluating the quality of remote education.

## Figures and Tables

**Figure 1:** Training results.

**Figure 2:** DANet-S structure.

**Figure 3:** Distance education quality assessment mode based on convolutional neural network.

The article "Construction of a Prediction Model for Distance Education Quality Assessment Based on Convolutional Neural Network" was published in 2022. Journal: Comput Intell Neurosci.

**Figure 4:** Comparison of the accuracy of distance teaching quality assessment.

**Figure 5:** Efficiency comparison of distance teaching quality assessment.

**Figure 6:** Prediction robustness of distance education quality assessment for three algorithms.

**Figure 7:** *F*1 value predicted by distance education quality assessment of three algorithms.

**Table 1:** The process of identifying data sources.

Step	Specific contents
Fit state established	Establish fit state in simulation environment
Data denoising	Clear wrong data
Data source exclusion	Exclude unreliable or marginal data sources
Algorithm choice	Select an algorithm for preparing data. Particularly the method that makes up the difference for the data deficiency

**Table 2:** Network error test results.

Training function name	dm	da	Dx	lm
Average network error	0.0014	0.0109	0.0041	0.0007

**Table 3:** Teaching quality evaluation index hierarchy.

Target layer	Criterion layer	Indicator layer
Teaching quality	Teacher teaching situation	T11 well prepared before class
		T12 The main points of the explanation are highlighted
		T13 link theory with practice
		T14 teacher-student interaction
		T15 modern teaching methods
		T16 focus on ability development
		T17 caring for students
		T18 teacher table
		T19 The overall effect of teaching is good
	Course information	T21 course content
		T22 course load

**Table 4:** Basic data.

Basic situation	Category	Frequency
Gender	Male	47
	Female	53

Used identity	Teacher	21
	Student	79

Academic area	Natural science	59
	Social science	41

Education level	Bachelor degree and below	57
	Graduate student or above	43

**Table 5:** The generality of distance teaching quality assessment model.

Course title	Evaluation accuracy/%	Modeling time/s
University English	95.23	22.61
Communication principle	94.62	23.53
Linear algebra	94.84	23.86
Engineering mechanics	93.65	22.47
University Chinese	95.13	26.95
Basic computer science	96.35	24.67
Machine learning	95.29	23.29

## Data Availability

The data used to support the findings of this study are included within the article.
